The article "Modulation of gut microbiota alleviates cerebral ischemia/reperfusion injury in rats by inhibiting M1 polarization of microglia" was published in 2023. Journal: Front Pharmacol.

# Modulation of gut microbiota alleviates cerebral ischemia/reperfusion injury in rats by inhibiting M1 polarization of microglia

**DOI:** 10.3389/fphar.2023.1123387

**Published:** 2023-05-09

**Authors:** Hai-Jun Li, Dan-Qing Li, Yu-Liang Zhang, Xiao-Fei Ding, Hai-Tao Gao, Ya Zhu, Jun Liu, Li-Xia Zhang, Jie Chen, Guang Chen, Ying Yu

**Affiliations:** ^1^ Department of Neurology, Taizhou Second People’s Hospital, Taizhou University, Taizhou, Zhejiang, China; ^2^ Department of Pharmacology, School of Medicine, Taizhou University, Taizhou, Zhejiang, China; ^3^ Department of Hygiene Toxicology, School of Public Health and Management, Wenzhou Medical University, Wenzhou, Zhejiang, China; ^4^ Laboratory Department, Municipal Hospital Affiliated to Medical School of Taizhou University, Taizhou, Zhejiang, China

**Keywords:** cerebral ischemia/reperfusion injury, gut microbiota, microglial polarization, fecal microbiota transplant, NF-κB–nuclear factor kappa B

## Abstract

Gut microbiota affects the gut–brain axis; hence, the modulation of the microbiota has been proposed as a potential therapeutic strategy for cerebral ischemia/reperfusion injury (CIRI). However, the role and mechanism of the gut microbiota in regulating microglial polarization during CIRI remain poorly understood. Herein, using a middle cerebral artery occlusion and reperfusion (MCAO/R) rat model, we evaluated changes in the gut microbiota after CIRI and the potential effects of fecal microbiota transplant (FMT) on the brain. Rats underwent either MCAO/R or sham surgery, and then they received FMT (started 3 days later; continued for 10 days). 2,3,5-Triphenyltetrazolium chloride staining, neurological outcome scale, and Fluoro-Jade C staining showed that MCAO/R induced cerebral infarction, neurological deficits, and neuronal degeneration. In addition, immunohistochemistry or real-time PCR assay showed increased expression levels of M1-macrophage markers—TNF-α, IL-1β, IL-6, and iNOS—in the rats following MCAO/R. Our finding suggests that microglial M1 polarization is involved in CIRI. 16 S ribosomal RNA gene sequencing data revealed an imbalance in the gut microbiota of MCAO/R animals. In contrast, FMT reversed this MCAO/R-induced imbalance in the gut microbiota and ameliorated nerve injury. In addition, FMT prevented the upregulation in the ERK and NF-κB pathways, which reversed the M2-to-M1 microglial shift 10 days after MCAO/R injury in rats. Our primary data showed that the modulation of the gut microbiota can attenuate CIRI in rats by inhibiting microglial M1 polarization through the ERK and NF-κB pathways. However, an understanding of the underlying mechanism requires further study.

## 1 Introduction

Ischemic stroke typically results from focal occlusion or arterial stenosis in the brain, and it poses a serious threat to the life of the affected individual (The Lancet Neurology, 2020). Ischemia/reperfusion injury is a pathological process associated with restoration of blood supply to the brain after a period of ischemia (Lin et al., 2016). Characteristics of ischemia/reperfusion injury include brain tissue necrosis, neurological dysfunction, and cognitive impairment (Jurcau and Simion, 2021). The molecular mechanism underlying the damage caused by cerebral ischemia/reperfusion injury is highly complex; however, it has been reported to involve oxidative stress, neuroinflammation, and apoptosis (Wu et al., 2020). In particular, neuroinflammation is a key factor in the ischemic cascade (Stoll and Nieswandt, 2019)—excessive inflammation can exacerbate cerebral ischemic injury (Werner et al., 2020). As a resident subset of immune cells in the brain, microglia exist as proinflammatory M1 or anti-inflammatory M2 functional phenotypes (Orihuela et al., 2016). Neuroinflammation caused by the aberrant polarization of microglia is an important mechanism underlying cerebral ischemia/reperfusion injury (Jurcau and Simion, 2021).

In recent years, there has been rapid progress in research regarding gut microbiota; the role of the gut microbiota in the occurrence and development of neuropsychiatric diseases is becoming clear (Bonnechère et al., 2022). Bidirectional communication within the gut–brain axis explains the potential role of the gut microbiota in the pathogenesis of neuropsychiatric diseases. The composition of the intestinal flora in patients with ischemic stroke and animal models of ischemic brain injury is significantly altered (Li et al., 2019). However, the mechanisms underlying the effects of the intestinal flora on cerebral ischemia/reperfusion injury remains unclear. The gut microbiota can modulate the physiology of microglia in the central nervous system; its presence is considered a prerequisite for the normal development and function of microglia (Wang Y. et al., 2018). Intestinal flora imbalance and microglial dysfunction have been observed to coexist in patients with neuropsychiatric diseases, suggesting a possible relationship between the intestinal flora and microglial state. The gut microbiota may be involved in the occurrence and development of cerebral ischemia/reperfusion injury. However, the role and mechanism of the gut microbiota in microglial polarization during cerebral ischemia/reperfusion injury remains poorly understood. In addition, the effects of microglia-mediated neuroinflammation on cerebral ischemia/reperfusion injury remain unclear. Therefore, integrative studies on the relationship between gut microbiota and microglia are urgently required. In the present study, we mimicked cerebral ischemia/reperfusion injury using the MCAO/R rat model and treated the rats with FMT for 10 days. At the end of experiment, we collected the rats’ rectal feces and brain tissues; afterward, we detected the gut microbiota profile, cerebral infarct area, neurological deficit, and M1 or M2 type gene expression profiles of microglia, to study the relationship between gut microbiota, microglia, and neuroinflammation.

## 2 Materials and methods

### 2.1 Animals

The animal study protocol was ethically approved by the Medical Ethics Committee of Taizhou University College of Medicine (Approval No. TZYX-2022-20221038). Experiments were performed on 8-week-old male Sprague–Dawley (SD) rats (weighing 300–300 g) obtained from Beijing Vital River Laboratory Animal Technology Co., Ltd. All the animals (*n* = 22; five rats per cage) were kept in a temperature and humidity-controlled environment with a 12-h light/dark cycle, temperature of 22°C–25°C, 50%-65% humidity, and free access to food and water. The rats were euthanized by exposure to 4% isoflurane followed by cervical dislocation.

### 2.2 Middle cerebral artery occlusion (MCAO)

Focal cerebral ischemia was induced by left MCAO using a protocol previously described, but with slight modifications (Stubbe et al., 2013; Li et al., 2020). Sixteen rats were first anesthetized with 1.5%–2% isoflurane v/v oxygen. The right external carotid artery (ECA), common carotid artery, and internal carotid artery (ICA) were all isolated. A 4-0 nylon suture 3 cm in length with a slightly enlarged and rounded tip was inserted from the ECA into the lumen of the ICA to block the MCA source. The distance was 17–20 mm from the tip of the suture to the bifurcation of the common carotid artery. Following 90 min of MCAO at 37°C, with anesthesia maintained throughout the period, reperfusion was performed by withdrawal of the suture until the tip cleared the lumen of the ECA. In the sham group, six rats underwent identical procedures but without insertion of the nylon monofilament.

### 2.3 Fecal microbiota transplant (FMT)

On day 3, after undergoing MCAO/reperfusion (MCAO/R0, the rats were randomized into the following treatment groups (six rats each group): 1) the antibiotic cocktail plus fecal microbiota transplant group, where the rats received a daily dose of 1.25 mg/L vancomycin, 2.5 mg/L amoxicillin, and 2.5 mg/L metronidazole by oral gavage for 3 consecutive days (days 3–5) to “delete” inherent flora from the intestine (Amorim et al., 2022), followed by FMT from days 6–15 and 2) the vehicle treatment group.

Fecal microbiota collected from the fresh feces of healthy SPF (Specific-pathogen-free) male SD rats (weight, 260–280 g) were transferred to a centrifuge tube containing PBS solution and centrifuged at 2,000 g for 15 min. The supernatant was discarded, and the pellet was washed with normal saline. This process was repeated to prepare a fecal bacteria transplantation suspension.

### 2.4 Profiling of the gut microbiota

Using a previously described protocol (Liang et al., 2022), rectal feces were processed for total DNA extraction via the cetyltrimethylammonium bromide/sodium dodecyl sulphonate method. DNA concentration and purity were monitored on 1% agarose gel before being diluted to 1 ng/μL using sterile water. Subsequently, 16 S ribosomal (r) RNA genes of distinct regions (16 S V3-V4) were amplified using a specific primer pair (forward: 5′-CCTAYGGGRBGCASCAG-3′; reverse: 5′-GGACTACNNGGGTATCTAAT -3′). All PCR reactions were performed using Phusion^®^ High-Fidelity PCR Master Mix (New England Biolabs, Inc.). Afterwards, equal volumes of 1X loading buffer (SYB green) were mixed with the PCR products and subjected to electrophoresis on 2% agarose gel for detection. Samples with bright main strips 400–450-bp long (16 S) and 100 to 400-bp long (ITS) were chosen for further experiments. PCR products were combined in equidensity ratios. The mixture of PCR products was then purified using Qiagen Gel Extraction Kit (Qiagen GmbH). Sequencing libraries were generated using TruSeq^®^ DNA PCR-Free Sample Preparation Kit (Illumina, Inc.), according to the manufacturer’s protocols, before the index codes were added. Library quality was assessed using Qubit^®^ 2.0 Fluorometer (Thermo Fisher Scientific, Inc.) and Agilent Bioanalyzer 2,100 system (Agilent Technologies, Inc.). Subsequently, the library was sequenced on an Illumina NovaSeq 6,000 platform (Illumina, Inc.), where 250 bp paired-end reads were generated. The raw tags were double-ended reads, which could be accessed through fastq join (v1.3.1; https://code.google.com/p/ea-utils/) and pear (v0.9.11). As the original sequence contained two primer sequences, Cutadapt (v1.18) was used to isolate the sequences without primers and cut out the fully sequenced primers from the reads. Q30. Usearch (version 11.0.667) with no ambiguous bases was used to cluster according to 97% similarity. We calculated alpha diversity was calculated using Mothur v1.42.1, beta diversity using the ‘vegan’ package in R, and pathway enrichment using the PICRUSt2 software package (https://github.com/picrust/picrust2) (Douglas et al., 2020).

### 2.5 2,3,5-Triphenyltetrazolium chloride (TTC) staining

The rats were rapidly anesthetized with isoflurane (1.5%–2%); afterwards, their brains were removed and frozen at −20°C for 5 min. Each brain was cut into five 2 mm slices and refrigerated at −20°C. The brain tissue sections were immersed in 1% TTC staining solution (Leagene Biotechnology) at 37°C for 20 min. The presence of infarction was determined by any area stained negative with TTC.

### 2.6 Neurological deficit assessment

Neurological deficit assessments were performed by investigators who were blinded to the experimental groups, as previously described (Wang J. et al., 2018). The following rating scale was used: i) 0, no deficit; ii) 1, failure to extend left forepaw; iii) 2, decreased grip strength of left forepaw; iv) 3, circling to left by pulling the tail; and v) 4, spontaneous circling.

### 2.7 Fluoro-Jade C (FJC) staining

According to the protocols of Biosensis Fluoro-Jade C (FJC) Ready-to-Dilute Staining Kit (cat. no. BSS-TR-100-FJT; Biosensis Pty, Ltd.), slides were incubated in a mixture of sodium hydroxide and 70% ethanol for 5 min, and washed in 70% ethanol for 2 min and thereafter, in distilled water for 2 min. Subsequently, the slides were incubated in 0.06% potassium permanganate (Sinopharm Chemical Reagent Co., Ltd.) solution for 10 min at room temperature; afterwards, they were rinsed in distilled water for 2 min. The slides were incubated in 0.0001% FJC for 10 min at room temperature, and then stained with 4′,6-diamidino-2-phenylindole (Beyotime Institute of Biotechnology) and protected from light. Subsequently, the slides were then rinsed three times with distilled water for 1 min each. After drying at 50°C–60°C for 5 min, the slides were cleared by immersion in xylene for 1 min and sealed with coverslips after DPX mountant was added. Using a blinded strategy, the slides were visualized via a fluorescence microscope (BX53; Olympus Microsystems, Inc.) The number of FJC-positive neurons (cells/field) were calculated in three sections per slice.

### 2.8 Histological analysis

For histological analyses, brain tissues were fixed in 4% paraformaldehyde/PBS solution for 24–48 h at room temperature. Subsequently, the tissues were dehydrated in an ascending ethanol gradient, cleared in toluene, and embedded in paraffin. In total, 5-µm paraffin sections were stained with hematoxylin & eosin (H&E) to assess overall cardiac morphology using an optical microscope (BX53; Olympus Microsystems, Inc.).

### 2.9 Immunohistochemistry and cell counting

Immunohistochemistry was performed on 30-μm free-floating sections. After deparaffinization, rehydration, antigen retrieval, neutralization of endogenous peroxidase, and blocking with 10% normal serum, the slices were incubated with primary antibodies such as anti-pERK (CST, Cat #4370S), anti-Arg (Proteintech, Cat #16001-1-AP), anti-NF-kB p65 (ABCAM, Cat #ab16502) at −4°C overnight. Thereafter, the slices were washed three times with PBS before secondary antibodies were added (anti-Rb IgG/HRP was obtained from Proteintech; the dilution rate was 1:1000). After incubation at room temperature for 1 h, the slices were washed three times with PBS and colored with 3,3′-diaminobenzidine. Finally, the slices were counterstained with H&E at room temperature. A microscope and ImageJ were used to analyze stained slices. Only brown color was considered positive marking regardless of color intensity.

### 2.10 Reverse transcription quantitative PCR (RT-qPCR)

Brain tissue samples were homogenized in TRIzol reagent (Invitrogen; Thermo Fisher Scientific, Inc.) Total RNAs were harvested using the TRIzol reagent, according to the manufacturer’s protocol, before reverse transcription was performed by the reverse transcription kit (Takara Biotechnology Co., Ltd.) to obtain the cDNA. The synthetized cDNA was amplified by qPCR using the following specific primers (Table 1).

**TABLE 1:** Primer list.

Gene	Primers	
	Forward	Reverse
IL-1β	CCA​CAG​ACC​TTC​CAG​GAG​AAT​G	GTG​CAG​TTC​AGT​GAT​CGT​ACA​GG
TNF-α	CTC​TTC​TGC​CTG​CTG​CAC​TTT​G	ATG​GGC​TAC​AGG​CTT​GTC​ACT​C
IL-6	AGA​CAG​CCA​CTC​ACC​TCT​TCA​G	TTC​TGC​CAG​TGC​CTC​TTT​GCT​G
iNOS	AAG​CAG​CAG​AAT​GAG​TCC​CC	CCT​GGG​TCC​TCT​GGT​CAA​AC
Arg-1	ACG​GAA​GAA​TCA​GCC​TGG​TG	GTC​CAC​GTC​TCT​CAA​GCC​AA
TGF-β	TAC​CTG​AAC​CCG​TGT​TGC​TC	CGG​TAG​TGA​ACC​CTG​CGT​TG
IL-4	CCG​TAA​CAG​ACA​TCT​TTG​CTG​CC	GAG​TGT​CCT​TCT​CAT​GGT​GGC​T
IL-10	TCT​CCG​AGA​TGC​CTT​CAG​CAG​A	TCA​GAC​AAG​GCT​TGG​CAA​CCC​A
GAPDH	GCA​CCG​TCA​AGG​CTG​AGA​AC	GCC​TTC​TCC​ATG​GTG​GTG​AA

The qPCR cycles were as follows: 95°C for 30 s (step 1), followed by 40 cycles of 95°C for 5 s and 60°C for 30 s (step 2), 95°C for 15 s, 60°C for 60 s, and 95°C for 15 s (step 3). Target gene expression level was calculated using the 2^−ΔΔCq^ method with the following formula: ΔΔCt = ΔCt sample−ΔCt control gene and wherein ΔCt = Ct target gene—Ct internal reference.

### 2.11 Statistical analysis

All statistical analyses were performed in GraphPad Prism version 8.0 (GraphPad Software, Inc.) Most statistical significances were tested by one-way ANOVA and Tukey’s test. Neurological deficits scores were analyzed using a non-parametric test. Results were expressed as means ± SEM, *n* = 6. *p* < 0.05 was considered to indicate a statistically significant difference.

## 3 Results

### 3.1 FMT decreases the cerebral infarct area and neurological deficit score induced by MCAO/R

The cerebral infarct area was detected by TTC staining of brain slices. There were no infarct lesions in the sham group; however, all treatment groups exhibited infarct lesions. We found that the percentage of infarct size in the brain tissues of rats in the MCAO/R group was approximately 32%. In contrast, healthy FMT conferred partial protection, with the percentage of infarct size in the brain tissues of rats in the MCAO/R + FMT group being approximately 24% (*p* = 0.001 vs. MCAO/R group; Figures 1A, B).

**FIGURE 1:** FMT alleviates cerebral infarction injury induced by middle cerebral artery occlusion/reperfusion. **(A)** Representative images of TTC staining in brain sections. The infarcted area according to TTC staining is shown in white. **(B)** Statistical analysis of the percentage cerebral infarction area in each group of rats. **(C)** Statistical analysis of the neurological deficit scores on a 5-point scale. The data are presented as the means ± SEM. Statistical analysis was performed using one-way ANOVA and Tukey test (*n* = 6). **(D)** Representative images of hematoxylin and eosin staining in brain tissues. FMT, fecal microbiota transplant; TTC, 2,3,5-triphenyltetrazolium chloride.

Neurological deficits were examined and scored on a 5-point scale. As shown in Figure 1C, compared with those in the sham group, rats in the MCAO/R model group manifested hemiplegia and their scores were significantly higher. With healthy FMT, the scores significantly decreased compared with those in the MCAO/R model group. Furthermore, H&E staining results showed more serious neurological damage in MCAO/R model, whereas healthy FMT blocked this process (Figure 1D).

### 3.2 FMT prevents ischemia/reperfusion-induced neuronal damage

To evaluate the effect of FMT on neuronal degeneration, we performed FJC staining of brain tissues. As shown in Figures 2A, B, the numbers of FJC-positive cells in the MCAO/R model group were significantly higher compared with those in the sham groups, whereas the numbers of FJC-positive cells were markedly lower in the FMT group compared with those in the MCAO/R model group.

**FIGURE 2:** FMT prevents ischemia/reperfusion-induced neuronal damage. **(A)** Representative images of FJC staining in brain tissues. **(B)** Statistical analysis of the number of FJC-positive cells in each group. The data are presented as the means ± SEM. Statistical analysis was performed using one-way ANOVA and Tukey test (*n* = 6). FMT, fecal microbiota transplant; FJC, Fluoro-Jade C.

### 3.3 FMT reverses the imbalance of gut microbiota induced by MCAO/R in rats

Using 16 S rRNA gene sequencing analyses, we characterized the microbial composition of the rectal fecal samples collected from rats 10 days after treatment. Microbial community bar plots showed that the microbiota composition of the genus and phylum was altered significantly (Figures 3A, B) after cerebral infarction. In terms of the microbial composition on a genus level, MCAO/R decreased the relative abundance of *Ligilactobacillus* from 56.21% to 14%, *Romboutsia* from 10.74% to 1.01% and HT002 from 22.75% to 5.68%; whereas it increased the relative abundance of *Escherichia-Shigella* from 0.43% to 16.49%, *Staphylococcus* from 0.01% to 2.15%, *Lactobacillus* from 6.29% to 26.38%, *Streptococcus* from 0.09% to 2.64%, *Akkermansia* from 0.17% to 18.74%, *Corynebacterium* from 0.26% to 2.00%, *Bacteroides* from 0.01% to 0.64%, *Bilophila* from 0.04% to 1.4%, and *Firmicutes*_unclassified from 0.02% to 0.29% in MCAO/R model rats compared with those in the sham control rats. Compared with the MCAO/R model group, FMT appeared to have partially reversed the imbalance (Figure 3A).

**FIGURE 3:** Configuration of gut microbiome diversity in each group of rats. **(A)** Genus levels. **(B)** Phylum levels.

On the phylum level, we analyzed the components and found that the relative abundance values of Proteobacteria (0.59%–17.14%), *Verrucomicrobiota* (0.17%–18.74%), *Actinobacteriota* (0.34%–2.06%), Bacteroidota (0.19%–1.16%), and *Desulfobacterota* (0.14 1.47%) were significantly increased in MCAO/R rats compared with those in the sham control rats. The relative abundance of *Firmicutes* (98.51%–59.40%) was significantly decreased in the MCAO/R group (Figure 3B). FMT prevented these changes at the phylum level induced by MCAO/R injury.

### 3.4 FMT inhibits MCAO/R-induced M1 polarization of microglia

Microglia function as the first line of defense in the brain; M2-to-M1 microglial shift during chronic inflammation following stroke has been reported to aggravate neuronal injury (Hu et al., 2012). Using immunohistochemistry and immunofluorescence, we detected the expression of iNOS and CD206 in brain tissues. As shown in Figure 4, the expression level of the M1-type marker iNOS was significantly increased in the MCAO/R model group compared with that in the sham group, whereas FMT prevented this type of M1 polarization (Figure 4A). In contrast, the expression level of the M2-type marker CD206 increased to a degree in the MCAO/R model group, but FMT further increased CD206 expression level (Figures 4B, C).

**FIGURE 4:** Fecal microbiota transplant reverses M2 to M1 microglia polarization induced by middle cerebral artery occlusion/reperfusion. **(A)** Representative images of inducible nitric oxide synthase immunohistochemical staining in brain tissues from each group. **(B)** Representative images of CD206 immunofluorescence staining in brain tissues from each group. **(C)** Statistical analysis of the numbers of CD206-positive cells in each group. Data were presented as the means ± SEM. Statistical analysis was performed using one-way ANOVA and Tukey test (*n* = 6).

We measured the mRNA expression levels of M1-type genes (IL-1β, IL-6, iNOS, and TNF-α; Figure 5A) and M2-type genes (Arg1, IL-4, IL-10, and TGF-β; Figure 5B) using RT-qPCR. Consistent with aforementioned results, expression levels of the M1 markers (IL-1β, IL-6, iNOS, and TNF-α) were higher in the tissues after MCAO/R, whereas FMT inhibited this increase. However, FMT potentiated an increase in the expression levels of Arg1, IL-10, IL-4, and TGF-β induced by MCAO/R. This suggests that M2-type microglia markers can promote the survival of neurons in normal and ischemic/hypoxic conditions.

**FIGURE 5:** Fecal microbiota transplant regulates the expression levels of M2/M1 microglia polarization genes. **(A)** mRNA expression levels of M1-type genes, IL-1β, IL-6, iNOS, and TNF-α, in brain tissues as detected using RT-qPCR. **(B)** mRNA expression levels of M2-type genes, arginase 1, IL-4, IL-10, and transforming growth factor-β, were measured using RT-qPCR. All expression levels were normalized to that of GAPDH. Data are presented as fold changes relative to the mRNA levels in sham group tissues. The data are presented as the means ± SEM. Statistical analysis was performed using one-way ANOVA followed by Tukey test (*n* = 6). FMT, fecal microbiota transplant; IL, interleukin; iNOS, inducible nitric oxide synthase; TNF, tumor necrosis factor; RT-qPCR, reverse transcription quantitative PCR.

### 3.5 FMT prevents MCAO/R injury-induced M2/M1 shift through the ERK and NF-κB pathways

M1-type gene expression is regulated by NF-κB (Streit et al., 2004) and MAPK signaling, and it plays an important role in cerebral ischemia/reperfusion injury (Fann et al., 2018). In the present study, we measured the protein expression levels of NF-κB and phosphorylated ERK in brain tissues after MCAO/R with or without FMT. As shown in Figure 6A, NF-κB expression level was found to be higher in the MCAO/R group than in the Sham group; however, but there was lower nuclear NF-κB staining in the MCAO/R + FMT group than in the MCAO/R group. Similarly, rat brain tissues from the MCAO/R group exhibited higher levels of ERK phosphorylation than that in the sham group. However, FMT inhibited the activation of ERK induced by MCAO/R (Figure 6B).

**FIGURE 6:** Representative images of rat brain tissues after phosphorylated extracellular-signal regulated kinase and nuclear factor-κB immunohistochemical staining. **(A)**, p-ERK staining; **(B)**, NF-κB staining.

## 4 Discussion

Gut microorganisms play a crucial role in regulating the development and outcomes cerebral ischemia/reperfusion injury (Malkki, 2016). In the present study, we mimicked cerebral ischemia/reperfusion injury using the MCAO/R model in rats, which resulted in clear changes in the gut microbiota profile. We analyzed gut microbiome composition by detecting rectal fecal samples of rats using 16 S ribosomal RNA (rRNA) gene sequencing. Compared with crypt content, rectal fecal samples can be collected more conveniently, making its collection more feasible in clinical practice. The present study showed that on a genus level, MCAO/R decreased the relative abundance of *Ligilactobacillus*, *Romboutsia*, and HT002. In contrast, the relative abundance values of *Escherichia-Shigella*, *Staphylococcus*, *Lactobacillus*, *Streptococcus*, *Akkermansia*, *Corynebacterium*, *Bacteroides*, *Bilophila,* and *Firmicutes*_unclassified increased compared with those in the sham control rats. On the phylum level, the relative abundance values of *Proteobacteria*, *Verrucomicrobiota*, *Actinobacteriota*, *Bacteroidota*, and *Desulfobacterota* increased in MCAO/R model rats compared with those in the sham control rats, whereas the relative abundance of *Firmicutes* significantly lower in the MCAO/R group.

The genus *Shigella* and *Staphylococcus*—belonging to the family *Enterobacteriaceae* and *Staphylococcaceae,* respectively—were previously found to promote cerebral ischemia/reperfusion injury (Kraemer et al., 2008; Rasmussen et al., 2009; Lee et al., 2021). *Shigella* and *Staphylococcus* bacterial cells invade M cells that are important for immune activation, which are phagocytosed by macrophages which subsequently undergo apoptosis, leading to inflammation (Rey et al., 2020). Seventy percent of the human body’s inflammatory and immune cells are localized in the gut, and these cells can migrate to the brain during cerebral ischemia injury, leading to poor outcomes in ischemia/reperfusion patients (Zhou et al., 2023).

Microglia are resident immune cells in the brain and mainly exist as the M1 or the M2 phenotype, in a manner where they can dynamically interconvert between the two phenotypes (Morrison and Filosa, 2019). Microglia have been found to activate and switch to the anti-inflammatory M2 phenotype during the acute phase of stroke, peaking at 3 days after stroke, which plays an important role in synaptic remodeling (Wicks et al., 2022). However, as the disease progresses, the aberrant activation of microglia by damaged neurons rapidly transforms microglia into the proinflammatory M1 phenotype, which in turn aggravates the disease (Hu et al., 2012; Kirkley et al., 2017). In the present study, we showed that expression levels of M1-type genes, IL-1β, IL-6, iNOS, and TNF-α, significantly increased 15 days after MCAO/R, whilst FMT prevented this increase. In contrast, the expression levels of M2-type genes, CD206, Arg1, IL-4, IL-10, and TGF-β, were further elevated by FMT in MCAO/R rats. These findings suggest that cerebral ischemia/reperfusion injury induces microglial polarization to M1, which worsens the extent of inflammation and neurotoxicity.

FMT involves the transfer fecal bacteria and other microbes from a healthy donor to another patient, which is an effective treatment method for treating certain bacterial infections (Liubakka and Vaughn, 2016). At present, alterations in the gut microbiota balance can lead to the onset of several diseases, such as Alzheimer’s disease (Angelucci et al., 2019), obesity (Patterson et al., 2016), diabetes (Patterson et al., 2016) and cancer (Xu J. Y. et al., 2021). Recent studies are increasingly focusing on the relationship between the gut microbiota-brain-gut axis and diseases of the nervous system (Sampson et al., 2016; Quigley, 2017). Xu et al. (2021) showed that ischemic stroke rapidly triggered gut microbiome dysbiosis with *Enterobacteriaceae* overgrowth, which in turn exacerbated brain infarction.

In the present study, FMT reversed this imbalance in the gut microbiota of animals with MCAO/R, which alleviated nerve injury. In addition, our results showed that FMT decreased the upregulation in NF-κB and ERK activity. Classical NF-κB is a key transcription factor involved in the regulation of cytokine production and serves as a major regulator of microglial inflammation (Zaghloul et al., 2020). The well-known downstream target genes of ERK/NF-κB signaling, IL-1β, IL-6, iNOS, and TNF-α, are also M1-type genes. They were found to be significantly increased following MCAO/R, whereas FMT prevented this upregulation.

Our primary data showed that gut microbiota imbalance triggers the abnormal polarization of microglia to the M1 type, which then mediates neuroinflammation and aggravates the injury induced by MCAO/R. The underlying mechanism is likely to be associated with the activation of ERK and/or NF-κB signaling. FMT could, therefore, attenuate these events and is a promising therapeutic method for cerebral ischemia/reperfusion injury.

## Data Availability

The original contributions presented in the study are included in the article/Supplementary Material, further inquiries can be directed to the corresponding authors.
